The article "Application of Cement-Based Carbon Fiber Material in Construction of Building Durability" was retracted in 2023. Reasons: signs of a paper mill; compromised peer review; unreliable results or conclusions.

# Application of Cement-Based Carbon Fiber Material in Construction of Building Durability

**DOI:** 10.1155/2022/3562209

**Published:** 2022-11-09

**Authors:** Qiuhong Li, Yinlong Li, Yong Zhang, Yongrui Han

**Affiliations:** School of Civil Engineering and Architecture, NanChong Vocational and Technical College, Nanchong, Sichuan 637000, China

## Abstract

In order to solve the problem of drying shrinkage of cement-based carbon fiber materials in the early stage of hardening, the author proposes the application of cement-based carbon fiber materials in the construction of building durability. The author uses a self-designed fast ring test method to test and study the drying shrinkage performance of cement-based carbon fiber materials in the early stage of hardening. The results showed that the addition of MP-I and MP-II fibers, which can significantly reduce shrinkage cracking in plastic concrete, has little effect on preventing the shrinkage and cracking of concrete in the early stage of hardening. Mixed with a certain amount of steel fiber, carbon fiber, MH-I, and MPH-I hardened anticrack fiber, all have a better effect on preventing early water loss and drying shrinkage of hardening. The MH-I and MPH-I hardening anticracking fibers have an economical and feasible dosage, and the early water loss shrinkage and crack reduction rates of concrete hardening are 71.2% and 79.0%, respectively. MH-I fibers have no anticracking effect in the plastic stage and are only suitable for shrinkage and crack prevention of concrete in the early stage of hardening, while MPH-I hardened anticrack fibers have a 100% crack-reducing effect in the plastic stage, it is an engineering fiber material that can simultaneously prevent the plasticity and early hardening of concrete from shrinkage and cracking. The application of MPH-I hardened anticrack fiber is of great significance to improve the quality of structural engineering.

## 1. Introduction

With the development of human society, the detection and evaluation of various large buildings has become a research hotspot of domestic and foreign experts. Concrete is the most important material in basic buildings such as civil and industrial, and its performance plays a very important role in the durability of buildings and the response to emergencies [1]. Cement mortar and concrete can be regarded as binary composite materials in which isolated aggregate particles are dispersed in a homogeneous medium; therefore, their related properties can be simulated by the related theory of binary system, in which there is an interface region in the range of 20–50 *μ*m on the aggregate surface whose structure and properties are different from that of the cement paste body, which is called the cement paste-aggregate interface transition zone.

Cement-based carbon fiber materials refer to cement-based composite materials that use cement mortar, cement slurry, or concrete as a binder and intermittent short fibers or continuous long fibers as reinforcing materials [2]. Adding a certain amount of fiber to cement mortar can not only improve the stiffness and toughness of concrete but also help the tensile strength, flexural strength, and toughness of cement-based composite materials, in addition, it can effectively inhibit crack propagation and improve the fluidity of nonforming materials, which is the most effective way to improve its performance. Generally speaking, the resistivity of ordinary cement-based composite materials is in the range of 104∼107 Ω·m under normal conditions, which is a kind of nonconductive material. Carbon fiber materials are widely used in various fields due to their electrical conductivity, thermal conductivity, controllability of surface morphology, low density, and low quality; this is also the main reason why it can become an ideal reinforcing fiber material [3]. However, due to the frequent agglomeration of carbon fiber materials, it is difficult to disperse in cement-based composite materials, studies have shown that adding dispersants or using ultrasonic technology can make them have better dispersibility in solution. Various studies have shown that doping carbon fiber materials into cement-based composites can effectively reduce or improve the electrical conductivity of their surfaces, in order to adapt to various environmental needs, and enhance its tensile strength and flexural strength [4, 5].

In recent years, with the development of science and technology, the quality of carbon fiber has been significantly improved, and the cost has also been significantly reduced, this has greatly increased the market demand for carbon fiber-reinforced cement-based composites. Due to the superior properties of carbon fiber-reinforced cement-based composites compared with other materials, they will be more widely used in civil engineering and other civil fields. The cement-based carbon fiber material is a composite material prepared by doping carbon fiber material in cement-based composite material, it has the advantages of high crack resistance, corrosion resistance, antistatic, wear resistance, and lightweight. The improvement of carbon fiber materials on cement-based composites mainly comes from its excellent mechanical properties and the use of the synergistic effect of the two materials to improve their overall mechanical properties [6, 7].

The physical, mechanical, and various physical and chemical properties of carbon fiber materials and cement-based composite materials are very different, in particular, the cement-based composite material has the characteristics of low bonding strength to the surface of many materials due to the transition zone of the cement paste-aggregate interface [8]. This characteristic will make the interface structure dominated by debonding failure on the bonding surface, and the addition of carbon fiber material will significantly improve this state. Cement-based composites modified by carbon fiber materials will show excellent compressive, tensile, impact resistance, and other characteristics, this also makes carbon fiber cement-based composites have good applications in many aspects [9].

## 2. Literature Review

With the progress of the times and the development of society, people have more requirements for cement, the most basic building material industry. As a composite material, cement-based carbon fiber material can effectively change its physical and chemical properties through the synergistic effect of carbon fiber materials and cement-based composite materials, so that it can be used in various environments. Although the agglomeration of carbon fiber materials in cement-based composites can be improved by adding dispersants, it is still the focus and difficulty of research to find auxiliary types that can improve or even eliminate the agglomeration phenomenon. Carbon fiber is a new type of material with high strength, large modulus, and excellent mechanical properties. The carbon content in it exceeds 95%, which is a microcrystalline graphite material obtained by carbonization and graphitization of organic fibers. Carbon fiber has many excellent properties, its specific gravity is less than 1/4 of that of steel, but its strength is higher than that of steel, and it has the characteristics of corrosion resistance and high modularity, it has good properties of not easy to creep, high temperature and fatigue resistance in the nonoxidizing environment [10, 11]. A composite material is a material with two or more different properties, including a material with new properties composed of physical or chemical methods, such as a material composed of reinforcing material and polymer matrix, cement-based carbon fiber material, in recent years, it has developed rapidly and is widely used in aerospace, machinery, electronics, chemical industry, and other fields.

Ahmad, H. S.et al tested the electromagnetic shielding effect of carbon fiber cement-based composites, adding carbon and carbon fiber to the cement-based composites, respectively, the results show that as the mass fraction of carbon black increases over 6%, the electromagnetic shielding effect of cement-based composites has been greatly improved [12]. Carbon fiber is a more effective additive than carbon, with the increase of carbon fiber content, the shielding effectiveness gradually increases, and the maximum electromagnetic shielding effect reaches 27 dB in the tested frequency range [13]. Carbon fiber cement-based composites not only have good applications in electromagnetic shielding but also have good applications in electrical conductivity. For example, when Gagnon, B. et al. doped carbon fiber materials into cement-based composites, the double infiltration phenomenon (involving fiber infiltration and cement slurry infiltration) was observed for the first time [14]. Experiments show that at a fixed volume fraction of carbon fibers in the slurry fraction, the electrical conductivity of the mortar decreases with an increasing sand/cement ratio.

Plastic shrinkage cracking and hardening shrinkage cracking of the concrete, in light of the rework caused by the direct impact on the appearance quality of the project during the construction stage, in the worst case, it will affect its impermeability, antifreezing, antichemical medium erosion, anticorrosion of steel bars and other properties, as a result, the service life of concrete is shortened and the maintenance and repair costs are increased. In China, the paving mileage of concrete pavement alone is nearly 10,000 km every year, once the pavement cracks, it will seriously affect the performance of the pavement, making it very difficult to repair and the cost is huge. Concrete shrinkage cracking is one of the main reasons for the above situation, at present, there are no technically and economically feasible measures to deal with this problem at home and abroad, therefore, the authors carried out research on the dry shrinkage cracking properties of cement-based carbon fiber materials and their anticracking measures, which is of great significance to improve the quality of structural engineering.

## 3. Methods

### 3.1. Experimental Raw Materials

The cement is Conch brand P. 0.42.5 grade ordinary Portland cement, the sand is medium sand with a fineness modulus of 2.60, the stone is a crushed stone of 5∼15 mm, the water is tap water, and the fibers are MP-I, MP-II, MH-I, and MPH-I anticracking engineering fibers produced by a company. The steel fiber is the cutting steel fiber produced by a steel fiber factory, and the carbon fiber is the PAN-based carbon fiber produced by a carbon factory.  Table 1 lists the physical and mechanical properties of the fibers used.

### 3.2. Experimental Method of Plastic Water Loss Shrinkage Cracking of Cement-Based Carbon Fiber Materials

The plastic water loss shrinkage cracking experiment of cement-based carbon fiber material adopts 914 mm × 610 mm × 19 mm wood mold, and the mortar is mixed according to the ratio of w (cement): w (sand): w (water) = 1.0 : 1.0 : 0.5 [15, 16].

### 3.3. Experimental Method of Drying Shrinkage Cracking in the Early Stage of Hardening of Cement-Based Carbon Fiber Materials

The experimental method of drying shrinkage cracking in the early stage of hardening of cement-based carbon fiber materials is as follows: the concrete is stirred for about 3 minutes according to the ratio of w (cement): w (sand): w (stone): w (water) = 1.0 : 0.5 : 0.5 : 0.5 (for other mortars, other materials are added at the same time), pouring in early hardening shrinkage cracking trial molds. The test piece is a cylindrical body with an inner diameter of 150 mm, a height of 150 mm, and a thickness of 20 mm, a steel cylindrical body with an outer diameter of 150 mm, a height of 150 mm, and a thickness of 30 mm is placed inside as a restraining body. After the specimen was formed, it was taken out after standard curing for 3 days, and the accelerated drying and dehydration shrinkage cracking experiment was carried out in a box with a temperature of 70 °C and a humidity of 20%, the temperature was heated up to 70 °C with a heating system of 10°C · h^−1^ and a constant temperature of 1 h, and then the temperature was kept constant. Measure the water loss rate of the specimen, observe whether there is cracking with the naked eye, and end the experiment when the water loss rate decreases to a roughly stable temperature (about 70°C constant temperature for 24°h). The crack width was determined by the JC-10 reading microscope produced by Precision Instrument Co., Ltd., and the crack length L_i_ was measured in sections according to the crack width d, according to the crack width weight Ai listed in Table 2, the following formula is used to calculate the crack weight value:

(1) $$\begin{array}{c} W=\sum A_{i}L_{i} \end{array}$$

where W reflects the total length of shrinkage cracking after early hardening, cm.

## 4. Results and Discussion

### 4.1. Effect of Fibers on Drying Shrinkage Cracking in the Early Stage of Hardening

Steel fibers were added at 0.2%, 1.0%, and 2.0% (volume fraction, the same below) of the concrete mixture, respectively, the weight value Wr of hardening shrinkage cracking relative to the standard concrete is shown in Table 3.

It can be seen from Table 3 that the low content of steel fiber not only has no crack reduction effect, but increases cracks by 51.2%, this is related to the defects of the steel fiber being self-heavy. Due to the low fiber content and the high water-cement ratio, when the slurry is relatively thin, the aggregate is easily affected by the steel fibers to sink and segregate, forming an uneven structure with a dense lower part and a sparse upper part. During the actual measurement, it was found that more cracks appeared in the upper part of the ring, and the upper cracks were wider and longer than the lower ones. When the fiber content is increased to more than 1.0%, due to the increase in the proportion of steel fibers in the concrete, a three-dimensional network structure is formed in the entire range of the specimen, which effectively exerts the advantages of high elastic modulus and high tensile strength of the fiber itself, the crack reduction effect is obvious. The 1.0% steel fiber content reduces the shrinkage cracking of the concrete ring by 83.3% in the early stage of hardening, while the 2.0% steel fiber concrete has no cracks at all.

### 4.2. Effect of Carbon Fiber on Drying Shrinkage Cracking in the Early Stage of Hardening

According to 0.125%, 0.25%, 0.5%, and 1.5% of the concrete mixture, carbon fiber is added, and the weight of the hardening shrinkage cracking is shown in Table 4.

It can be seen from Table 4 that the shrinkage cracking of concrete gradually decreases with the increase of carbon fiber content. Compared with the benchmark concrete, 0.125% and 0.25% carbon fiber concrete reduces cracks by 36.0% and 41.5%, respectively, when the carbon fiber content is greater than 0.5%, cracks can be completely eliminated. This should also be attributed to the characteristics of carbon fiber's high elastic modulus. However, in the actual molding process, the construction performance of the concrete after adding carbon fiber is greatly reduced, and only a small amount of water-reducing agent can be added to increase the fluidity to facilitate molding. The high manufacturing cost of carbon fiber also limits its application in practical engineering.

### 4.3. Effect of Engineering Anticracking Fibers on Drying Shrinkage Cracking in the Early Stage of Hardening

MP-I, MP-II, MH-I, and MPH-I engineering anticracking fibers were used to study their effects on drying shrinkage cracking in the early stage of concrete hardening.  Table 5 lists the weight values of drying shrinkage cracking in the early stage of hardening of fiber-reinforced concrete with different contents.

It can be seen from Table 5 that 0.10% of MP-I and MP-II fibers were added, although their crack reduction rates for plastic shrinkage cracking were as high as 79.3% and 99.5%, respectively; however, the reduction rate of shrinkage cracking in the early stage of hardening of concrete is only 8.1% and 0%, respectively, indicating that due to the small elastic modulus of the fiber, it can only play a role in plastic crack prevention; After adding 0.125% MH-I fiber, the shrinkage cracking of concrete in the early stage of hardening was reduced by 71.2% and adding 0.25% MPH-I fiber concrete, the shrinkage cracking in the early stage of hardening is reduced by 79.0%, the difference between the two is that the MPH-I type engineering anticrack fiber has both plasticity and anticrack effects in the early stage of hardening, its plastic crack reduction effect will be described later.

### 4.4. Effect of Hardened Anticracking Fibers on Plastic Shrinkage Cracking

The plastic shrinkage cracking experiment was carried out with the above-mentioned hardening shrinkage anticracking fiber under the condition of low dosage, and the total weight value of plastic shrinkage cracking obtained by the measurement is listed in Table 6.

It can be seen from Table 6 and Figure 1 that steel fibers have little effect on preventing plastic shrinkage cracking; The plastic crack prevention effect of carbon fiber is very good, but its disadvantage is that it is expensive; Although MH-I fiber has an obvious effect on preventing shrinkage cracking in the early stage of concrete hardening, it has no anticracking effect on plastic shrinkage cracking, on the contrary, the plastic shrinkage cracking weight value is more than doubled compared with the benchmark mortar. Therefore, it is only suitable for crack prevention after hardening. Although the content of MPH-I fiber is doubled compared with that of MH-I, its plastic crack reduction effect is 100% compared with the benchmark mortar and combined with its hardening crack prevention effect, it can reach 79.0%, overall, it shows a dual anticracking effect on the plastic stage and early hardening of cement concrete, and its price is much lower than that of carbon fiber materials, making it an excellent anticracking fiber material [17]. The difference in plastic cracking between the two fibers may be related to their fiber parameters, in MH-I fibers, there are more short fibers below 5 mm, while in MPH-I fibers, there are more long fibers above 5 mm. Since the bonding strength between fibers and cement slurry is very weak in the plastic stage, longer fibers can significantly improve the bonding force between fibers and cement slurry, so the plastic crack reduction rate is significantly improved; In the hardening stage, because the bonding strength between the fiber and the cement stone has been significantly improved, the shorter fiber can also play a better anticracking effect, and the effect of the fiber length on the bonding force is weakened, so the fiber length is in the hardening crack reduction rate, the effect of length is also weakened accordingly, and this phenomenon needs further research in the future.

### 4.5. Effect of Hardened Anticracking Fibers on Mechanical Properties of Cement-Based Materials

Table 7 lists the effect of 0.25% MPH-I hardening anticracking fiber on the mechanical properties of cement mortar and concrete [18–20].

It can be seen from Table 7 that after adding MPH-I fiber with plasticity and hardening dual anticracking effect in cement mortar and concrete, there is no obvious adverse effect on its fluidity and mechanical strength.

## 5. Conclusion

The author proposes the application of cement-based carbon fiber materials in the construction of building durability and tests the drying shrinkage performance of cement-based carbon fiber materials in the early stage of hardening. The test result indicates, adding 0.10% of MP-I and MP-II fibers, which can significantly reduce the shrinkage and cracking of plastic concrete, has little effect on preventing the shrinkage and cracking of concrete in the early stage of hardening. Since the bonding strength between fibers and cement slurry is very weak in the plastic stage, longer fibers can significantly improve the bonding force between fibers and cement slurry, so the plastic crack reduction rate is significantly improved. In the hardening stage, because the bonding strength between fibers and cement stone has been significantly improved, shorter fibers can also play a better anticracking effect, and the effect of fiber length on the bonding force is weakened, therefore, the effect of fiber length on the hardening and crack reduction rate is also weakened, and this phenomenon needs further research in the future.

## Figures and Tables

**Figure 1:** Effect of hardened anticracking fibers on plastic shrinkage cracking.

**Table 1:** Physical and mechanical properties of fibers.

Fiber type	Density/(g · cm^−3^)	Diameter /*μ*_m_	Length/mm	Elastic modulus/GPa	Tensile strength/MPa	Elongation/%
Carbon fiber	1.61	7	19	251.0	2500	1.1
Steel fiber	7.91	561^1^	34	201.0	984	3.4
MP-I MP-II fibers	0.92	33	14	3.3	400	30.1
MH-I fibers	2.61	15	5 ~ 20	200.1	3000	8.1
MPH-I fibers	1.31	5	6 ~ 18	37.1	1360	7.1

(1) is the equivalent diameter.

**Table 2:** Fracture width weight Ai Table.

*d*/mm	0 < *d* < 0.05	0.05 < *d* < 0.10	0.10 < *d* < 0.20	0.20 < *d* < 0.30	0.30 < *d* < 0.40	0.40 < *d*
*A*_*i*_	0.024	0.053	0.140	0.230	0.340	0.420

**Table 3:** Effect of steel fiber content on drying shrinkage cracking in the early stage of hardening.

Type of concrete	*W*/cm	*W*_r_/%
Benchmark concrete	2.11	100.2
Mixed with 0.2% steel fiber reinforced concrete	3.22	151.4
Mixed with 1.0% steel fiber reinforced concrete	0.33	16.5
Mixed with 2.0% steel fiber reinforced concrete	0.01	0.11

**Table 4:** Effect of carbon fiber content on drying shrinkage cracking in the early stage of hardening.

Type of concrete	*W*/cm	*W*_r_/%
Benchmark concrete	4.01	100.01
Mixed with 0.125% carbon fiber concrete	2.55	64.01
Mixed with 0.25% carbon fiber concrete	2.35	58.51
Mixed with 0.5% carbon fiber concrete	0.01	0.1
Mixed with 1.5% carbon fiber concrete	0.01	0.1

**Table 5:** Effects of engineering fibers on drying shrinkage cracking in the early stage of hardening.

Type of concrete	*W*/cm	*W*_r_/%
Benchmark concrete	3.09	100.0
0.10% *M* P–I fiber reinforced concrete	2.84	91.9
Mixed with 0.10% MP-II fiber-reinforced concrete	3.09	100.0
Mixed with 0.125% MH-I fiber concrete	0.89	28.8
0.25% MPH-I fiber-reinforced concrete	0.65	21.0

**Table 6:** Effect of hardened anticracking fibers on plastic shrinkage cracking.

Mortar type	*W*/cm	*W*_r_/%
Benchmark mortar	102.2	100.1
Mixed with 0.2% steel fiber mortar	103.1	100.8
Mixed with 0.125% carbon fiber mortar	2.91	2.81
Mixed with 0.125% MH-I fiber mortar	258.5	253.2
Mixed with 0.25% MPH-I fiber mortar	0.01	0.01

**Table 7:** Effects of MPH-I fibers on the physical and mechanical properties of mortar concrete.

Type of material	Slump or subsidence	Age/d	Flexural strength/MPa	Compressive strength/MPa
Benchmark concrete	6	3	2.35	21.21
		7	2.52	29.71
		28	2.44	37.12

Add 0.25% MPH-I fiber concrete	5	3	2.56	21.91
		7	2.51	27.71
		28	2.43	37.02

Benchmark mortar	8.20	3	5.46	29.71
		7	7.19	36.12
		28	8.12	48.72

Mixed with 0.25% MPH-I fiber mortar	6.10	3	6.18	29.61
		7	7.53	36.21
		28	8.48	49.01

## Data Availability

The data used to support the findings of this study are available from the corresponding author upon request.
